RETRACTED

# The Immunoregulation Effect of Alpha 1-Antitrypsin Prolong β-Cell Survival after Transplantation

**DOI:** 10.1371/journal.pone.0094548

**Published:** 2014-04-10

**Authors:** Yun Wang, Hong-Jie Yan, Shu-Yan Zhou, Yun-Shuang Wang, Hui Qi, Chun-Yan Deng, Fu-Rong Li

**Affiliations:** 1 Department of Cardiac Surgery, General Hospital of Ningxia Medical University, Yinchuan, PR China; 2 The Key Laboratory of Stem Cell and Cellular Therapy, The Second Clinical Medical College (Shenzhen People's Hospital), Jinan University, Shenzhen, PR China; 3 Shenzhen Institution of Gerontology, Shenzhen, PR China; University of Michigan Medical School, United States of America

## Abstract

Islet transplantation has considerable potential as a cure for diabetes. However, the difficulties that arise from inflammation and the immunological rejection of transplants must be addressed for islet transplantation to be successful. Alpha 1-antitrypsin (AAT) inhibits the damage on β cells caused by inflammatory reactions and promotes β-cell survival and proliferation. This protein also induces specific immune tolerance to transplanted β cells. However, whether the expression of AAT in β cells themselves could eliminate or decrease immunological rejection of transplants is not clear. Therefore, we established a β cell line (NIT-hAAT) that stably expresses human AAT. Interestingly, in a cytotoxic T lymphocyte (CTL)-killing assay, we found that hAAT reduced apoptosis and inflammatory cytokine production in NIT-1 cells and regulated the Th1/Th2 cytokine balance in vitro. In vivo transplantation of NIT-hAAT cells into mice with diabetes showed hAAT inhibited immunological rejection for a short period of time and increased the survival of transplanted β cells. This study demonstrated that hAAT generated remarkable immunoprotective and immunoregulation effects in a model of β cell islet transplantation for diabetes model.

## Introduction

Type 1 diabetes results from autoimmune destruction of insulin-producing pancreatic β cells, and is characterized by hyperglycaemia due to reduced insulin secretion. Apoptosis is the main mode of pancreatic β cell death in the development of diabetes [1]. Since the implementation of the Edmonton protocol in 2000 [2], islet transplantation has become one of the most promising options to cure Type 1 diabetes. Islet transplantation has been evaluated as a procedure that could enable patients to regain physiological glucose control, yet the immunologic tolerance protocol that accompanies this procedure excludes diabetogenic corticosteroids, resulting in the exposure of grafted cells to an unopposed inflammatory environment [3]. Similar to the process of islet injury during transplantation, the autoimmune response that is directed toward islets in a type 1 diabetic individual appears to overlap with several immune processes that occur during allograft rejection [4]. Autoimmunity and immunological rejection are the two major side effects resulting from islet transplantation. Thus, there is increasing motivation to identify an islet-protective antiinflammatory immune-modulating agent that is safe for use.

RETRACTED

Alpha 1-antitrypsin (AAT) is a key serine protease inhibitor [5]. The protein has anti-inflammatory, anti-leukocyte migratory, anti-thrombotic, and anti-apoptotic effects [6]–[9], and also exerts cytoprotective effects upon islets in vitro [8], [10]. As expression of AAT sharply rises in response to inflammation, AAT may function to limit the duration and magnitude of inflammation [11]. Furthermore, short-term AAT treatment restores euglycemia and self-tolerance to islets in overtly T1D nonobese diabetic (NOD) mice [12]. In addition, AAT promotes insulin secretion of islet cells in mice [13]. Therefore, we hypothesized that a transplant of β cells expressing AAT would have a low chance of immunological rejection due to the anti-inflammatory and anti-apoptotic functions of AAT. Essentially, these AAT-expressing cells could induce specific immune tolerance to the transplant.

In the present study, pDsRed–hAAT was transfected into NIT-1 cells, and a stable cell line was generated. By conducting cytotoxic T lymphocyte (CTL)-killing assays and cell transplantations into diabetic mice, we found that hAAT expression reduced immunological rejection of the inflammatory reactions against the β-cell transplantation. Our results indicate that hAAT can exhibit an immune protective effect on transplanted β cells.

## Materials and Methods

### Plasmid construction

The pBS–RSV–hAAT plasmid was donated by Prof. Andre Lieber (University of Washington, U.S.A). The region encoding hAAT was amplified and subcloned into the eukaryotic expression vector pDsRed-N111 (donated by Prof. Lu Zhigang, Peking University Shenzhen Graduate School, China) to generate the pDsRed–hAAT vector.

### Construction of the stable hAAT-NIT-1 cell line

NIT-1 cells (a kind gift from Prof. Li Fangping, Sun Yat-Sen University, China), an insulin-producing insulinoma cell line, derived from non-obese diabetic (NOD) mice prone to autoimmune diabetes [14] were used as a cell model system. These cells were expanded in 24-well tissue culture plates in Dulbecco's modified Eagle's medium (DMEM; Sigma, St. Louis, MO, USA) with 10% FCS (Gibco, CA, USA). Liposome 2000 (Invitrogen, Carlsbad, CA, USA) was utilized to transfect pDsRed–hAAT or pDsRed mock-vector into the NIT-1 cells respectively. Seventy-two hours after the transfection, G418 (350 µg/mL, Sigma) was added to the medium for selection. Low-dose G418 (175 µg/mL) was subsequently applied to generate cells stably expressing the construct. The 10^th^ and the 40^th^ generation of the NIT-hAAT cell line were collected and lysed. Western blotting was conducted to validate that hAAT was expressed at the protein level. The hAAT levels from cultured supernatant samples (72 h) at passage 10 and passage 40 (5×10^5^ cells/mL)were determined by Human Alpha 1-Antitrypsin ELISA(Immunology Consultants Laboratory, Newberg,OR, USA).

RETRACTED

### Mice

BALB/c mice (8 weeks old) were provided by the Experimental Animal Center of Guangdong Province. The mice were kept in the SPF Animal Laboratory (Experimental Animal Center of the Second Clinical Medicine College, Jinan University). This study was carried out in strict accordance with the recommendations in the Guide for the Care and Use of Laboratory Animals of the Second Clinical Medical College (Shenzhen People's Hospital), Jinan University. The protocol was approved by the Committee on the Ethics of Animal Experiments of the Second Clinical Medical College, Jinan University. All surgery was performed under sodium pentobarbital anesthesia, and all efforts were made to minimize suffering.

### Collection of lymphocytes

Sixty BALB/c mice, divided into three groups with 20 animals per group, were injected intraperitoneally with 5×10^6^ NIT-1 cells, 5×10^6^ NIT-vector cells and 5×10^6^ NIT-hAAT cells respectively at the first day and the tenth day. Twenty BALB/c mice were injected intraperitoneally with 5% Physiological saline (control group). At day 20, all mice from each group were sacrificed. The spleens were mashed to release single cells, and then red blood cells were lysed. The cells were later washed twice with RPMI 1640. The cells were filtered through a 200-mesh nylon net, and the lymphocytes concentration was adjusted to 1×10^6^ cells/mL.

### One-way mixed lymphocyte multiplication experiment

The lymphocytes from each group described above were utilized as the responder cells in a mixed lymphocyte reaction (MLR). NIT-1, NIT-Vector and NIT-hAAT cells were plated on a 12-well culture plate. When the cell concentration reached approximately 5×10^5^ cells/well, 1 mL of 30 mg/mL mitomycin C was added to each well, and the cells were incubated in the dark for 30 min. These cells were later used as the stimulator cells for the MLR. The ratios between the responder cells and the stimulator cells were 5∶1, 10∶1, 20∶1, and 50∶1. The cells were cultured in 5% CO_2_ at 37°C for 72 h. The cell counting kit-8 (CCK-8, Dojindo,Japan) was utilized according to the manufacturer's instructions to determine the number of cells in each well. The stimulation index (SI) of the responder cells was calculated according to the following equation: SI = (OD value of experimental well – OD value of blank well)/(OD value of negative control well – OD value of blank well). Three holes were analyzed for each group based on the negative control and blank wells.

RETRACTED

### Measurement of inflammatory cytokines

After seven days of mixing the culture at the ratio of 10∶1 of 5×10^6^ lymphocytes and mitomycin-based NIT-1,NIT-vector and NIT–hAAT cells in each group, the cultured supernatant was obtained and preserved at −80°C for later analysis. Mouse IFN-γ and IL-4 ELISA kits (Neobioscience, China) were utilized to determine the cytokine content of the supernatants. The absorbance was measured at 450 nm, and the cytokine levels were calculated based on the standard curve. Three different supernatants were analyzed for each sample.

### Determination of apoptosis

MLR with a ratio of 10∶1 of lymphocytes to NIT-1, NIT-vector and NIT–hAAT cells were allowed to proceed for seven days, and then the lymphocytes were removed. The NIT-1, NIT-vector and NIT–hAAT cells were collected and digested with pancreatin without EDTA. The cells concentration was adjusted to 1×10^6^ cells/mL, and 100 µL of the cells suspension were subsequently mixed with 5 µL of Annexin V-FITC and 1 µL of PI. The cells were incubated in the dark for 30 min and were washed twice with PBS. The number of cells undergoing apoptosis was determined by flow cytometry(BD Biosciences,Franklin Lakes, NJ, USA).

### Real-time quantitative PCR for CRP, IL-1β, IL-6 and IL10 mRNA

MLR with a ratio of 10∶1 of lymphocytes to NIT-1,NIT-vector and NIT-hAAT cells were allowed to proceed for seven days, and mRNA was extracted from the lymphocytes and reverse transcription was carried out with 1 µg of RNA. Real-time quantitative PCR was performed as previously described [15]. The following sequence-specific primers were used: CRP Forward: 5′-GGATTGTAGAGTTCTGGATTG-3′; CRP Reverse: 5′-TCACCCTGTGCTTTATAGTTC-3′; IL-1β Forward: 5′-GACGTTCCCATTAGACAACTGC-3′; IL-1β Reverse: 5′-GGTATAGATTCTTTCCTTTGAGGC-3′; IL-6 Forward: 5′-GACTTCCATCCAGTTGCCTTCT-3′; IL-6 Reverse: 5′-CCAGTTTGGTAGCATCCATCAT-3′; IL-10 Forward: 5′-TCCTTGGAAAACCTCGTTTG-3; IL-10 Reverse: 5′-CTTCAATTGCTTCCCAAGGA-3′; β-actin Forward: 5′-TACACCCAGGAAAGACAGCAACC-3′; and β-actin Reverse: 5′-CTCCTCGAAGACCTTCTCACAACCA-3′.

### Induction of diabetes in mice

Thirty BALB/c mice were injected intraperitoneally with a 2% STZ solution (170 mg/kg). The mice were later fed a high-sugar and high-fat diet. Diabetes was monitored by measurement of blood glucose concentration from the tail vein using a blood glucose device (Roche Accu Check III, Roche, Basel, Switzerland). Mice with non-fasting blood glucose 300 mg/dl for 3 consecutive days were considered as onset of diabetes.

RETRACTED

### β Cell transplantation

There was no difference of immune response between NIT-1 and NIT-vector cells in vitro, therefore, the diabetic BALB/c mice were randomly divided into three groups: (1) NIT-hAAT Group (n = 15), in which 1.5×10^7^ NIT-hAAT cells were injected under the left kidney capsule; (2) NIT-1 Group (n = 15), in which 1.5×10^7^ NIT-1 cells were injected under the left kidney capsule; and (3) Diabetes group (n = 15), where 0.1 mL of PBS was injected under the left kidney capsule. In addition, 10 normal BALB/c mice were used as control group.

### β-cell functionality after the transplantation

The tails of the BALB/c mice were cut for blood collection at 4:00 p.m. every day after the transplantation. A MediSense Optium blood glucometer and the paper disk method were utilized to test the non-fasting blood glucose concentration for 36 consecutive days. At the 30^th^ day, the left kidney was removed. A glucose tolerance test was conducted on the 14^th^ and 28^th^ days after transplantation. Briefly, the mice that underwent fasting for 6 h to 8 h were given an intraperitoneal injection of 2 g/kg glucose in saline. Blood was collected at 0, 15, 30, 60, 90 and 120 min to measure the blood sugar concentration. Additionally, on the 7^th^, 14^th^, 21^st^, and 28^th^ days after the transplantation, 0.5 mL of blood was collected from each mouse periorbitally. The serum was preserved at −20°C after centrifugal separation. ELISA (Mercodia, Sweden) were performed to determine the insulin and C-peptide levels in the serum.

### Pathological observation

At 14 and 28 days after the NIT-hAAT and NIT-1 cells were transplanted, three mice from each group were selected, and their left kidneys were collected. The tissue was fixed with 10% formaldehyde and embedded in paraffin. The tissue was cut into 5-µm sections and stained with HE. Under a 400× optical microscope, ten fields of visions were randomly chosen to record the number of infiltrating white blood cells in transplantation site.

### Fluorescence immunocytochemistry

At 28 days after the NIT-hAAT and NIT-1 cells were transplanted. The left kidneys tissue was collected, fixed with 10% formaldehyde and embedded in paraffin. The tissue was cut into 5-µm sections and incubated with rat anti-mouse insulin antibody (Zymed Laboratories), rabbit anti-human AAT(Abcam, Cambridge,UK) antibody overnight at 4°C. Tissue were further incubated with FITC-labeled goat anti-rat polyclonal antibody (Jackson ImmunoResearch) and PE-labeled donkey anti-rabbit (Rockland) at 37°C for 1 hour. Tissues were washed with 1×PBS three times. The tissues were observed under fluorescent microscope (ECLIPSE TE2000-U,Nike, Germany).

RETRACTED

### Statistical analysis

Comparisons between groups were analyzed by a two-sided *t* test or an ANOVA for experiments with more than two subgroups. The results are presented as the mean ± SEM.

## Results

### Generation of the NIT–hAAT cell line

In vitro expression of hAAT was examined by western blot. Untransfected NIT-1 cells and NIT-vector cells did not express hAAT; however, NIT-hAAT cells did express hAAT. No significant difference exists in protein expression between cells at passage 10 and passage 40. NIT-hAAT cells maintained stable expression of hAAT in vitro (Figure S1). The hAAT levels from cultured 72 h supernatant concentration at passage 10 and passage 40 (5×10^5^ cells/mL) were 355.33±22.79 µg/mL and 340.33±20.55 µg/mL, respectively.

### Immunoregulation effects of hAAT

#### One-way mixed lymphocyte multiplication experiment

NIT-1,NIT-vector and NIT-hAAT cells were treated with mitomycin C and used as stimulator cells in an MLR. Proliferation of lymphocytes co-cultured with the NIT-hAAT cells was greatly inhibited compared with those cultured with NIT-1 cells or NIT-vector (P<0.05). The inhibitory effects were enhanced as the ratio of NIT–hAAT to lymphocytes increased, demonstrating a dose–dependent effect (Figure 1). At the ratio of 10∶1, the effects presented a significant difference (P<0.01). The lymphocyte amplification ability of the NIT-1 group and NIT-vector group were remarkably better (P<0.01, P<0.05) compared with that of the control group and the NIT–hAAT group.

**Figure 1:** hAAT has protective and immunoregulation dual effects analysed by CTL assay. The effects of hAAT on a β islet cell line were examined via an extended CTL assay in vitro (n = 3). BALB/c mice were immunized twice with NIT-1 or NIT-vector or NIT–hAAT cells, and the splenocytes were collected. These splenoctyes were used as responder cells in a 7 day MLR, while NIT-1 or NIT-vector or NIT–hAAT cells pretreated with mitomycin C were used as stimulator cells. An in vitro CTL assay was later performed using NIT-1 or NIT-vector or NIT–hAAT cells as target cells. Target cells cultured with unprimed splenocytes were utilized as control cells. The stimulation index (SI) of NIT-1 primed lymphocytes co-cultured with NIT-1 or NIT-vector or NIT–hAAT cells (A).The stimulation index (SI) of NIT-vector primed lymphocytes co-cultured with NIT-1 or NIT-vector or NIT–hAAT cells (B), The stimulation index (SI) of NIT-hAAT primed lymphocytes co-cultured with NIT-1 or NIT-vector or NIT–hAAT cells (C). *P<0.05.

RETRACTED

#### Th1 and Th2 cytokine levels

The Th1 cytokine (IFN-γ) and Th2 cytokine (IL-4) levels in the supernatants of the lymphocyte-NIT-1 cell, NIT-vector, NIT-hAAT co-cultures were determined by ELISA. The results demonstrate that the levels of IFN-γ were significantly reduced and the levels of IL-4 were significantly elevated in cultures containing NIT-hAAT cells compared with those containing NIT-1 cells and NIT-vector cells (P<0.05). However, NIT-1-primed lymphocytes or NIT-vector-primed lymphocytes co-cultured with NIT-1 cells or NIT-vector did not exhibit significantly different levels of cytokines compared with NIT-hAAT-primed lymphocytes co-cultured with NIT-hAAT cells. (P>0.05; Table 1).

**Table 1:** Comparison of concentration of interferon (IFN)-γ and interleukin (IL)-4 in lymphocytes immunized by NIT-1, NIT-vector and NIT–hAAT cells (pg/mL,Mean±SD. n = 3).

	IFN-γ(Th1)			IL-4(Th2)		
Group	NIT-1	NIT-vector	NIT-hAAT	NIT-1	NIT-vector	NIT-hAAT
	lymphocytes	lymphocytes	lymphocytes	lymphocytes	lymphocytes	lymphocytes
NIT-1	218.3±4.9	222.5±3.2	196.1±1.8*	22.8±3.7	23.2±2.7	24.2±4.8*
NIT-vector	223.6±5.1	219.3±4.1	202.1±2.2*	24.6±4.2	27.8±3.4	26.8±4.1*
NIT-hAAT	41.8±3.5**	42.3±4.1**	33.5±5.8**	45.4±2.6**	46.5±2.7**	52.1±3.25**
Control	182.1±6.4	188.1±7.2	164.6±5.2	28.2±0.8	30.7±6.1	32.2±7.2

*P<0·05, NIT-1, NIT-vector group versus Control group;

**P<0·01 NIT-hAAT versus Control, NIT-1 and NIT-vector group. No significant difference between the NIT-1 and NIT-vector groups was observed(P>0.05). No significant difference between the NIT-1primed lymphocytes or NIT-vector primed lymphocytes and the NIT–hAAT primed lymphocytes was observed(P>0.05).

#### Expression of CRP, IL-1β,IL-6 and IL-10 mRNA

The IL-10 mRNA levels in the splenocytes collected from mice that received a NIT–hAAT cell transplant, as detected by real-time quantitative PCR, were significantly enhanced compared with that from mice that received NIT-1 cells or NIT-vector (P<0.05). However, the expressions of CRP,IL-1β and IL-6 mRNA of the inflammatory factors were decreased (P<0.05) (Figure 2). CRP, IL-1β, IL-6 and IL-10 mRNA levels were not significantly different between the NIT-1 and NIT-vector groups, indicating that hAAT inhibits the expression of the inflammatory gene through in vivo adjustment of related cytokine levels.

**Figure 2:** The expression of CRP, IL-1β, IL-6 and IL-10 mRNA was determined by real-time PCR(n = 3). Mice were immunized twice with NIT-1 or NIT-vector or NIT–hAAT cells, and the splenocytes were collected and co-cultured for 7 days with NIT-1 or NIT-vector or NIT–hAAT cells pretreated with mitomycin C. CTL assay was subsequently performed using NIT-1 or NIT-vector or NIT-hAAT cells as target cells in vitro. CRP mRNA levels(A), IL-1β mRNA levels (B), IL-6 mRNA levels (C), IL-10 mRNA levels (D). *P<0.05,**P<0.01.

RETRACTED

#### Detection of apoptosis

Seven days after the mixed culturing of NIT-1-primed or NIT-vector-primed or NIT–hAAT -primed lymphocytes and NIT-1 or NIT-vector or NIT–hAAT cells treated with mitomycin, flow cytometry was performed to analyze the mixed culture cells. The apoptosis of the NIT-1 cells and NIT-vector cells in the mixed culture containing NIT–1-primed or NIT-vector primed lymphocytes showed a significant increase (37.6±1.1%,32.5±2.1%)(Figure 3A,B). The apoptosis of the NIT-1 cells and NIT-vector cells in the mixed culture containing NIT–hAAT-primed lymphocytes was lower (12.9±0.4%, 14.3%±1.1%)(Figure 3C,D) (P<0.01). The apoptosis of the NIT–hAAT cells in the mixed culture containing NIT-1-primed and NIT-vector primed lymphocytes was lower (10.1±0.9%, 9.5±0.9%)(Figure 3E,F). However, the apoptosis of the NIT–hAAT cells was the lowest in the NIT–hAAT -primed lymphocytes (8.6%±1.3%) (Figure 3G)(P<0.01).

**Figure 3:** The apoptosis of NIT-1,NIT-vector and NIT-1-hAAT cells were analyzed by flow cytometric(n = 3). Apoptosis of NIT-1 and NIT-vector cells (A) mediated by NIT-1 primed lymphocytesp; Apoptosis of NIT-1 and NIT-vector cells (B) mediated by NIT-vector-primed lymphocytes; Apoptosis of NIT-1(C),NIT-vector(D) mediated by NIT-hAAT primed lymphocytes. Apoptosis of the NIT–hAAT cells mediated by NIT-1-primed(E) and NIT-vector (F)primed lymphocytes;.Apoptosis of the NIT–hAAT cells(G)mediated by NIT–hAAT -primed lymphocytes.

### Pancreatic functionality after the β-cell transplantation

#### Blood glucose levels and weight changes of the diabetic mice

NIT-1 or NIT–hAAT cells were transplanted to under the left kidney capsule of the diabetic mice. The blood sugar levels of the mice in each group were tested every three days (Figure 4A). On the 3^rd^ day after transplantation, the blood sugar levels of the NIT-1 and NIT–hAAT groups mice decreased sharply. The blood sugar concentration of the mice in the NIT-1 group increased at the 15^th^ day, the blood sugar concentration increased to 300 mg/dL. At the 30^th^ day after the removal of the left kidney, the blood sugar concentration did not exhibit obvious changes. The mice in the NIT–hAAT group maintained a normal blood sugar level up to 30 days. On the 30^th^ day after transplantation, upon the removal of the left kidney, the blood sugar level of the mice increased significantly and reached the standard level of diabetes. It showed that the NIT–hAAT cells could secrete insulin. The weights of the mice in the NIT–hAAT group steadily increased over time, while the weights of the mice in the NIT-1 group and the untreated diabetic group gradually decreased (Figure 4B).

RETRACTED

**Figure 4:** Transplantation of NIT–hAAT cells into STZ-treated diabetic mice. NIT-1 or NIT–hAAT cells were transplanted into diabetic mice. After transplantation, the blood sugar level, body weight, glucose tolerance, and insulin and C-peptide concentrations were monitored. (A) Blood sugar levels of the recipients (n = 10). (B) Changes in the body weight of the recipients (n = 10). (C,D) GTT at 14 d (c) or 28 d (d) after transplantation (n = 5). (E) In vivo glucose-stimulated insulin secretion in the recipients (n = 5). (F) In vivo C-peptide levels in the recipients (n = 5). *P-value <0.05,**P-value <0.01 compared with the diabetic group.

**Figure 5:** Pathological HE staining and immunostaining of the left kidneys after transplantation. NIT-1 group at 14 d and 28 d after transplantation. Fourteen days after the transplantation, only a small number of transplanted NIT-1 cells remained in the kidneys. No transplanted NIT-1 cells were observed after 28 d, showing that the cells occurred fibrosis(A, B). NIT–hAAT group at 14 d and 28 d after transplantation, Fourteen days after transplantation, most of transplanted NIT–hAAT cells were still visible in renal capsule. After 28 days, there were no significant changes in the numbers of infiltrating inflammatory cells and a number of the transplanted NIT–hAAT cells were still present in the renal capsule(C,D). (scale bars, 200 µm). Immunostaining was performed at 28 d after transplantation NIT-hAAT cells under the kidney capsule. After rehydration, sections were incubated with anti-insulin and anti-hAAT antibodies. Insulin and hAAT at 28 d after transplantation are shown(E,F,G). (scale bars, 50 µm).

#### Sugar tolerance test

At 14 days after transplantation, the mice were given an injection of glucose, and blood sugar levels were tested at several time points after the injection. Fifteen minutes after the glucose injection, the blood sugar levels of the mice in the NIT–hAAT group decreased quickly, whereas that of the NIT-1 and the diabetic group declined slightly (Figure 4C). When the glucose tolerance test was conducted 28 d after the transplantation, the mice in the NIT–hAAT group controlled their blood sugar levels, as we noted on the 14^th^ day after transplantation. However, the blood sugar levels in the NIT-1 and untreated diabetic groups mice did not decrease significantly in the times tested after the glucose injection (Figure 4D). These data indicated that the NIT-hAAT transplantation resulted in the presence of living β cells that were capable of regulating blood sugar levels.

RETRACTED

#### Insulin and C-peptide analysis

The insulin and C-peptide levels in the serum were increased three days after transplantation from the NIT-hAAT group mice and remained elevated throughout the periods tested. These levels were significantly higher compared with those from the untreated diabetic group (P<0.01). Three days after the transplantation, the insulin and C-peptide levels in the serum from the NIT-1 group mice were increased but stabilized after 14 days(P<0.05). Thereafter, the insulin and C-peptide levels gradually declined. On the 21^st^ day after transplantation, no significant difference was observed in the diabetic group (P>0.05). (Figure 4E and 4F).

### Histological

At 14 d and 28 d after cell transplantation, the left kidneys from mice in each group were stained with HE, and the pathological changes in the transplant sites were analyzed (Figure 5A–D). Fourteen days after the transplantation, only a small number of transplanted NIT-1cells remained in the renal capsule. No transplanted cells were observed after 28 d, showing that the cells occurring fibrosis. In contrast, fourteen days after transplantation, most of transplanted cells were still visible in renal capsule from mice in the NIT–hAAT group. There were significantly fewer infiltrating inflammatory cells in the NIT-hAAT group (14±2.9 cells) compared with the NIT-1 group (31±10.98 cells; P<0.01). After 28 days, there were no significant changes in the numbers of infiltrating inflammatory cells in the NIT-hAAT group (16±3.6 cells), and a number of the transplanted cells were still present in the renal capsule. Immunostaining was performed at 28 d after transplanted NIT–hAAT cells under the kidney capsule. The expression of transplanted NIT–hAAT group like insulin (green) and hAAT (red) in tissuse was investigated by immunofluorescence(Figure 5E,F,G). The NIT-1 group was not found to have positive expression of these proteins (data not shown).

## Discussion

NIT-1 is a NOD-derived β cell line and maintains the characteristics of primary β cells, such as the capability for secretion of insulin, NIT-1 cells are a well-validated cell model for the study of type 1 diabetes [14]. Recently, various studies suggested that AAT possesses qualities that are favorable for islet graft survival [8], [13], [16]. In particular, our group studied the improvement attributes of AAT for autoimmunity and allograft rejection in beta cell transplantation.In present study, It is the first in the field to explore AAT-expressing beta-cells as targets of an immune response. NIT-1 cells were transfected with a vector encoding hAAT to generate a NIT–hAAT stable cell line. pDsRed–hAAT is a 55-kb plasmid that holds the entire human AAT sequence, including exons and introns, and the ability to self-replicate without integrating into the genome [17]. The expression of hAAT was verified by western blot. The NIT–hAAT cell line continued proliferating and maintained hAAT secretion up to the 40^th^ passage of the cells.

RETRACTED

In Cytotoxic T lymphocyte (CTL) experiment in vitro, NIT–hAAT,NIT-vector and NIT-1 cells were co-cultured with CTLs from the same mice that had previously been treated with NIT–hAAT, NIT-vector and NIT-1 cells. The CTLs that were co-cultured with NIT–hAAT cells proliferated significantly less than those co-cultured with NIT-1 cells and NIT-vector. Furthermore, compared with the NIT-1 group and NIT-vector group, the CTLs co-cultured with NIT-hAAT cells secreted significantly lower levels of Th1 cytokines (IFN-γ) (P<0.05), and significantly higher levels of Th2 cytokines (IL-4). Compared with the cells in the NIT-1 and NIT-vector cultures, the IL-10 mRNA levels in CTLs co-cultured with NIT-hAAT cells were significantly elevated (P<0.05), while the levels of CRP, IL-1β and IL-6 mRNA were decreased (P<0.05). These mediators were reported to cause islet graft failure via antigen-independent inflammation and correlate with poor transplant outcome [18]–[20].Thus, the ability of hAAT to diminish inflammatory mediators in the graft tissue may provide the basis for the diminished alloimmune response and prolonged islet graft survival. C reactive protein (CRP) has been proposed as a marker of systemic inflammation [21]. CRP and other inflammatory factors are closely related, once the inflammation reaction initiated, CRP level increased. Furthermore, IL-10 is a pleiotrophic immunomodulatory cytokine that functions at different levels of the immune response [22]. Especially, IL-10 induces anergy of T cells by efficiently inhibiting their proliferation and cytokine production [23], [24]. The expression of IL-10 mRNA plays a key role in anti-inflammatory event, so the expression of inflammatory factors CRP, IL-1β and IL-6 mRNA were decreased.

The percentage of NIT-hAAT cells undergoing apoptosis was at its lowest level when NIT-hAAT-primed CTLs were co-cultured with NIT-hAAT cells (P<0.05), indicating that hAAT protected the NIT-1 cells from apoptosis. In agreement with our data, it has been demonstrated that hAAT inhibited damage to β cells by decreasing the levels of inflammatory cytokines, such as IFN-γ and IL-1β [25]. Recent study demonstrated that treatment with AAT protects β-cells against apoptosis through inhibition of caspase-3 activity in a dose-dependent manner [26]. Moreover, hAAT can directly inhibit caspase-3 activation in β cells and thus can function as an anti-apoptotic agent [27]. IL-4 is Th2-type cytokine that promotes Th0 to Th2 differentiation and inhibits Th0 to Th1 differentiation, thereby adjusting the Th1/Th2 cytokine balance. In our study, the NIT-hAAT cells promoted the production of IL-4; therefore, AAT could induce the production of Th2 cells, which would reduce the amount of Th1 cytokines produced. This protein also inhibits the expression of several inflammatory factors. The findings of this study also indicate that co-culture of NIT-hAAT- or NIT-vector or NIT-1-primed CTLs with NIT-hAAT cells caused reduced apoptosis of the NIT-hAAT cells. Taken together, these findings indicate that AAT has a role in immunosuppression [28].

RETRACTED

There was no difference of immune response between NIT-1 and NIT-vector cells in vitro.To examine the effect of AAT in vivo, NIT-1 or NIT-hAAT cells were transplanted onto the left kidney of diabetic mice. In mice that received NIT-hAAT cells, the blood sugar levels were significantly reduced three days after the transplantation, and these low levels were maintained until the 30^th^ day. After the removal of the left kidney, the blood sugar concentration rapidly increased and the mice developed hyperglycemia. In the NIT-1 transplantation group, the blood sugar levels of the mice were decreased three days after the transplantation, but after twelve days, the levels increased significantly. We observed that on the 14^th^, 21^st^, and 28^th^ days after transplantation, the insulin and C-peptide levels of the mice in the NIT–hAAT group were higher than those in the untreated diabetic and NIT-1 groups (P<0.05). Moreover, the weights of the mice in the NIT–hAAT group increased compared with those of the mice in the untreated diabetic and NIT-1 groups. The glucose tolerance tests and pathology also suggest that hAAT improves the survival of NIT-1 cells and lessens inflammatory infiltrates. In another islet transplantation study, Lewis et al. found that AAT hinders the infiltration of neutrophils, granulocytes, and macrophages into the transplanted tissue [8]. The cuff-shaped Treg cellular layer was formed around the transplant; These cells expressed Treg-related genes, such as Foxp3, TGF-β, and CTLA-4. Walters et al. discovered a similar protective cellular layer around the transplant that reduced inflammatory infiltration and extended the lifespan of the transplant [29]. Given that the beta cell line used in this study originates from the NOD/LT mice, immunological rejection was observed after the transplantation. Forced expression of AAT by transplanted NIT-1 cells demonstrated that islet cells can exhibit immunoprotective abilities and inhibit immunological rejection for a short time. By increasing IL-4 production, the Th1 and Th2 cell balance was skewed toward Th2, which inhibited inflammation and reduced the immunological rejection of the islet β cell transplantation. Thus, the lifespan of these transplanted β cells was extended. However, the in vivo mechanisms by which hAAT causes immunosuppression, induces immune tolerance, and maintains the survival of the islet cells need further investigation [30].

RETRACTED

In summary, an AAT-expressing β cell line was established and used for transplantations in diabetic mice. In vitro MLR experiments demonstrated that AAT can regulate immune functions and exhibits immunoprotective effects on islet cells. When NIT-hAAT cells were transplanted into diabetic mice, immunoregulation effect was observed, and transplant rejection was partially inhibited.

## Supporting Information

Figure S1 **hAAT expression was confirmed by Western blot assay.** 1. NIT-1 cells transfected with the vector containing the hAAT gene, 2. NIT-1 cells transfected with the empty vector.
(TIF)
